This article has been retracted.

# Effects of Metoprolol Succinate Combined with Entresto on Cardiac Function Indexes and Coagulation Function in Patients with Congestive Heart Failure

**DOI:** 10.1155/2022/9765884

**Published:** 2022-05-21

**Authors:** Yuanyuan Ding, Zufa Wei, Jian Li, Ling Zhu

**Affiliations:** ^1^Hubei Province Huangshi Puren Hospital Cardiovascular Medicine, 435002, China; ^2^Audit Office of Huangshi Central Hospital, Hubei Province, China

## Abstract

**Objective:**

To investigate the effects of metoprolol succinate combined with Entresto (Sacubitril Valsartan Sodium Tablets) on cardiac function and coagulation function in patients with congestive heart failure (CHF).

**Methods:**

About 120 patients with CHF treated from April 2018 to April 2021 were enrolled in our hospital. The patients were arbitrarily assigned into control group and study group. The control group was cured with metoprolol succinate sustained-release tablets, and the study group was cured with metoprolol succinate sustained-release tablets combined with Entresto. The curative effect, cardiac function, vascular endothelial function, oxidative stress, and coagulation function were compared.

**Results:**

First of all, we compared the general data, and there exhibited no difference in age, sex, course of disease, hypertension, coronary heart disease, diabetes, atrial fibrillation, and other general data (*P* > 0.05). Second, we compared the clinical efficacy. The effective rate of the study group (98.33%) was higher (90.00%) (*P* < 0.05). There exhibited no significant difference in cardiac function indexes before treatment, but after treatment, LVEF increased, LVESD and LVEDD decreased, LVESD and LVEDD in the study group were lower, and LVEF in the study group was higher (*P* < 0.05). Before treatment, there exhibited no significant difference in vascular endothelial function. However, the levels of CGRP and ET increased and the level of NO decreased, and the level of NO in the study group was lower, while the levels of CGRP and ET in the study group were higher after treatment (*P* < 0.05). There exhibited no significant difference in oxidative stress indexes before treatment, however, the levels of GSH-Px and SOD increased and the levels of MDA decreased after treatment, while the level of MDA in the study group was lower, while the levels of GSH-Px and SOD in the study group were higher (*P* < 0.05). Finally, we compared the indexes of blood coagulation function. There exhibited no significant difference before treatment, but after treatment, the levels of APTT, PT, and FIB decreased, and the levels of APTT, PT, and FIB in the study group were lower (*P* < 0.05).

**Conclusion:**

Clinical practice demonstrated that LVESD and LVEDD decreased and LVEF increased after treatment with Entresto combined with metoprolol in CHF patients, which can effectively facilitate cardiac function and vascular endothelial function, reduce oxidative stress reaction, and improve blood coagulation indexes, suggesting that Entresto combined with metoprolol can improve ventricular remodeling with good safety.

## 1. Introduction

In recent years, cardiovascular disease has become one of the most serious diseases affecting human survival. Heart failure, as the end-stage manifestation of a variety of cardiovascular diseases, occupies a very important position in cardiovascular diseases [1]. Congestive heart failure (CHF) is a syndrome in which cardiac structure or function is abnormal for various reasons, resulting in impaired ventricular filling and ejection function, resulting in cardiac output that is difficult to meet the metabolic needs of the body, and resulting in a series of complex clinical manifestations [1]. At present, the total population of CHF is large worldwide. According to the epidemiological survey, the prevalence rate of CHF in developed countries is 1-2%, and the prevalence rate of heart failure in adults aged 35-74 in China is 0.9% [2]. A previous epidemiological study on hospitalized patients in Hong Kong indicated that the total incidence of CHF was 0.7 ppm 1000 [1–3]. In recent years, the average life expectancy has also been extended, and the problem of aging has become increasingly prominent. For example, the incidence and comorbidity of various chronic diseases such as coronary heart disease (CHD), hyperlipidemia, diabetes, and chronic kidney disease are significantly increased [4]. These diseases may directly or indirectly lead to the occurrence and development of CHF [4]. Heart failure brings a heavy burden to the society and the family; therefore, it is very indispensable for the prevention and treatment of CHF [5].

Nowadays, metoprolol succinate is often employed in the clinical treatment of CHF. Metoprolol succinate is a selective *β*1-receptor blocker, which attaches importance to the control of hypertension and CHD, however, the clinical efficacy of metoprolol succinate alone when treating CHF needs to be enhanced [6]. In recent years, with the advent of drugs such as angiotensin receptor/enkephalin inhibitor (ARNI), there has been a great breakthrough in the treatment of CHF. As a kind of ARNI drugs, Entresto (Sacubitril Valsartan Sodium Tablets) are mainly composed of sacubitril and valsartan at 1 : 1. They can block angiotensin II receptor and inhibit enkephalin through LBQ657, the metabolite of sacubitril valsartan, which have beneficial effects on relaxing blood vessels, preventing and reversing cardiovascular remodeling and promoting urinary sodium excretion [7]. Meanwhile, previous studies have indicated that Entresto may also be effective in the fight against myocardial fibrosis, antisympathetic nervous system activity, inhibition of antidiuretic hormone release, improvement of myocardial relaxation and vagus nerve tension, and antimyocardial hypertrophy [8, 9]. For patients with CHF, studies have indicated that ACEI and ARB play a certain part in improving symptoms and reducing hospitalization rate [10]. Most of the treatment for CHF is symptomatic treatment [11]. In 2012, a phase II clinical trial PARAMOUNTHF study of Entresto was published. It was found that Entresto reduced BNP in patients with CHF at 12 weeks of treatment compared with valsartan in the control group and indicated a decrease in left atrial volume (LAV) and an improvement in cardiac function classification at 36 weeks of treatment compared with the control group [12]. Considering that natriuretic peptide is a strong predictor of poor cardiovascular prognosis in patients with CHF, the results of this study also lead researchers to expect that Entresto can benefit patients with heart failure [12]. However, as a new drug, the dosage and efficacy of Entresto in clinical application of various types of CHF are not clear, and the clinical efficacy of Entresto combined with metoprolol succinate when treating CHF is worthy of further exploration. Therefore, this study conducted an observational study on patients with CHF who were treated with Entresto and metoprolol succinate sustained-release tablets combined with Entresto in our hospital to evaluate the efficacy of this drug in clinic, in order to assist the better clinical application of Entresto to optimize the treatment of patients with CHF.

## 2. Patients and Methods

### 2.1. Demographic Information

A total of 120 patients with CHF treated from April 2018 to April 2021 were enrolled in our hospital. The patients were arbitrarily assigned into control group and study group. In the control group, the age was 36-77 years old, and the course of disease was 2-14 years, while in the study group, the age was 36-78 years old, and the course of disease was 2-13 years. There exhibited no statistical significance in the general data (see Table 1). This study was permitted by the Medical Ethics Association of our hospital, and written informed consent was obtained from all patients.

Inclusion criteria: the diagnostic criteria of heart failure: according to the 2018 Chinese guidelines for the diagnosis and treatment of heart failure [13], the classification and diagnostic criteria of chronic heart failure are as follows: (1) heart failure with decreased ejection fraction- (HFREF-) combined with the patient's history, symptoms, and signs of heart failure; if the patient's LVEF is less than 40%, it is diagnosed as HFREF. (2) Heart failure with preserved ejection fraction- (HFPEF-) if the patient has a history, symptoms, and signs of heart failure; if the patient's LVEF ≥ 50% and natriuretic peptide are elevated, at least one of the following items is satisfied: (i) left ventricular hypertrophy and/or left atrial enlargement and (ii) cardiac diastolic dysfunction; excluding the patient's symptoms caused by nonheart disease, the patient is diagnosed as HFPEF.

Exclusion criteria: (1) history of vascular edema; (2) severe stenosis of bilateral renal arteries; (3) symptomatic hypotension (systolic blood pressure < 95 mmHg); (4) severe liver damage (Child Pugh grade C); (5) biliary cirrhosis; (6) cholestasis; (7) pregnant and lactating women; (8) serum potassium > 5.4 mmol/L; (9) severe renal insufficiency (serum creatinine > 221umol/L (2.5 mg/dl) or eGFR < 30 ml/(min 1.73 m^2^); (10) malignant tumor; (11) history of allergy to ARB, ACEI, or ARNI drugs or similar chemical drugs; and (12) cardiac valvular disease.

### 2.2. Treatment Methods

The control group was given metoprolol succinate sustained-release tablets (manufacturer: AstraZeneca Pharmaceutical Co., Ltd.; Chinese medicine standard: J20150044) treatment, 23.75~47.50 mg can be added according to the recovery of the disease dose, but the single dose should not exceed 190 mg once per day.

The study group was treated with Sacubitril Valsartan Sodium Tablets (manufacturer: Beijing Novartis Pharmaceutical Co., Ltd.; Chinese Medicine Standard: J20190001) on the basis of the control group, 50~100 mg/twice per day. Both groups were treated continuously for 14 days.

### 2.3. Observation Index

#### 2.3.1. General Information

Access to patient-related case data, record all enrolled patients' age, sex, course of disease, hypertension, coronary heart disease, diabetes, atrial fibrillation, and other general data.

#### 2.3.2. Clinical Efficacy Evaluation

The clinical effects were compared. The criteria are as follows: significant effect: dyspnea, fatigue, lung rale, cough, jugular vein anger, and other symptoms basically disappeared, arrhythmia decreased by more than 90%, cardiac function improved by 2 or more grades; effective: dyspnea, fatigue, lung rale, cough, jugular vein anger, and other symptoms improved, arrhythmia decreased by 70-89%, and cardiac function improved by 1 grade. Ineffective: dyspnea, fatigue, lung rale, cough, jugular vein anger, and other symptoms do not change or aggravate. Total effective rate = (number of effective cases + number of effective cases)/total number of cases × 100%.

#### 2.3.3. Cardiac Function Index

The cardiac function indexes left ventricular ejection fraction (LVEF), left ventricular end-systolic diameter (LVESD), and left ventricular end-diastolic diameter (LVEDD) were compared before and after treatment. Siemens ACUSONX150 color Doppler ultrasound system was employed for detection.

#### 2.3.4. Vascular Endothelial Function Index

The indexes of vascular endothelial function calcitonin gene-related peptide (CGRP), nitric oxide (NO), and endothelin (ET)) were compared before and after treatment. CGRP and ET were detected by enzyme-linked immunosorbent assay (ELISA). Griess's reagent (Griess) was employed to detect NO.

#### 2.3.5. Oxidative Stress Index

The indexes of oxidative stress, containing glutathione peroxidase (GSH-Px), superoxide dismutase (SOD), and malondialdehyde (MDA), were compared before and after treatment. GSH-Px was detected by colorimetry, and SOD was detected by ELISA, then, MDA was detected by thiobarbituric acid method.

#### 2.3.6. Blood Coagulation Index

The coagulation indexes were compared before and after treatment, APTT: activated partial prothrombin time, PT: prothrombin time, and FIB: fibrinogen. The blood samples of patients were collected, and APTT, PT, and FIB were detected by automatic coagulation analyzer.

#### 2.3.7. Incidence of Adverse Reactions

Statistics on the incidence of adverse reactions between the two groups.

### 2.4. Statistical Analysis

SPSS 22.00 was adopted to process the relevant data in this study and complete the relevant statistical analysis. Meanwhile, the quantitative data should be in accordance with the normal distribution, represented by the mean ± standard deviation$\bar{x}\pm s$. The independent samples used between different groups were mainly completed by *t*-test. Paired *t*-test was employed to compare the data before and after treatment. *χ*^2^ test or corrected *χ*^2^ test was used to complete the test of qualitative data, and the percentage (%) was employed to express the results of qualitative data. *P* < 0.05 indicated that there exhibited statistical difference.

## 3. Results

### 3.1. Comparison of Demographic Data

First of all, we compared the general data, there exhibited no significant difference in age, sex, course of disease, hypertension, coronary heart disease, diabetes, atrial fibrillation, and other general data (*P* > 0.05). All the results are shown in Table 1.

### 3.2. Comparison of Clinical Efficacy

Second, we compared the clinical efficacy, and the effective rate of the study group (98.33%) was higher compared to the control group (90.00%) (*P* < 0.05). All the results are indicated in Figure 1.

### 3.3. Comparison of Cardiac Function Indexes

Next, we compared the cardiac function indexes. There exhibited no significant difference before treatment, however, the LVEF increased, LVESD and LVEDD decreased, and the LVESD and LVEDD of the study group were lower compared to the control group after treatment, while LVEF was higher compared to the control group (*P* < 0.05). All the results are shown in Table 2.

### 3.4. Comparison of Vascular Endothelial Function Indexes

Then, we compared the indexes of vascular endothelial function, there exhibited no significant difference before treatment, of note, after treatment, the levels of CGRP and ET increased and the levels of NO decreased, and the level of NO in the study group was lower, while the levels of CGRP and ET in the study group were higher (*P* < 0.05). All the results are indicated in Table 3.

### 3.5. Comparison of Oxidative Stress Indexes

Next, we compared the oxidative stress indexes, there exhibited no significant difference before treatment, however, the levels of GSH-Px and SOD increased and the levels of MDA decreased, and the level of MDA in the study group was lower after treatment, while the levels of GSH-Px and SOD in the study group were higher (*P* < 0.05). All the results are indicated in Table 4.

### 3.6. Comparison of Coagulation Function Indexes

Finally, we compared the indexes of blood coagulation function, there exhibited no significant difference before treatment, but after treatment. The levels of APTT, PT, and FIB decreased, and the levels of APTT, PT, and FIB in the study group were lower (*P* < 0.05). All the data results are indicated in Table 5.

### 3.7. Comparison of the Incidence of Side Effects between the Two Groups

Finally, we compared the incidence of adverse reactions. The incidence of side effects in the control group is 11.67%. The incidence of side effects in the study group is 3.33%, the study group was lower than the control group (*P* < 0.05). All the data results are indicated in Figure 2.

## 4. Discussion

CHF is a common cardiovascular disease in clinic, which often occurs in the middle-aged and elderly stage, with the characteristics of long course of disease, complex etiology, and various complications [1]. CHF has adverse effects on the health of tens of millions of people around the world and is regarded as the fastest growing cardiovascular disease with high incidence and high cost of treatment [2]. The relevant study implicates that the onset and development of CHF are closely related to various factors, and the key mechanism lies in the excessive activation of neuroendocrine system and cytokines, leading to gradual myocardial remodeling and continuous progress of CHF [14]. In the actual classification of CHF, the key to death in these patients depends on the relevant indicators of the left ventricle (LV) of CHF [15]. Patients with CHF can be treated with antiplatelet drugs, statins, diuretics, cardiotonic agents, and so on, among which metoprolol succinate is a commonly used drug in clinic [16]. Related research results indicate that metoprolol succinate can reduce sympathetic excitability, reduce myocardial oxygen consumption, and dilate blood vessels [17]. Metoprolol succinate can reduce blood pressure and heart rate. However, metoprolol succinate alone is not effective in the treatment of CHF [16].

The advent of Entresto (Sacubitril Valsartan Sodium Tablets) plays a potential part in the treatment and prognosis of CHF [18]. Through the persistence of many parties, the listing of Entresto has opened a new way to the treatment of CHF. The components of Entresto include equal proportion of sacubitril and valsartan. From acute to chronic phase, a number of important clinical trials have been published, containing the PARADIGM-HF study, the TRANSITION study, and the PIONEER-HF study [19]. Based on these findings, the first-line treatment of patients with ejection fraction retention heart failure (HFPEF) is determined to be Entresto, which was included in “European and American Heart failure guidelines,” “2018 Chinese Heart failure guidelines,” and “2019 European Heart failure Association expert consensus” [20]. In addition, the highest blood concentration can be achieved at 1.5-4.5 h after oral administration, the blood drug value can be maintained in the patient's body after 3 days, and the bioavailability is excellent [21].

Studies have confirmed that Entresto can also reduce enkephalinase activity [22]. Combination with metoprolol succinate in the treatment of CHF can give full play to their vasodilation effect, directly relax arteriole smooth muscle and reduce cardiac load, helping patients improve cardiac function [23]. Entresto is a new type of double-effect compound preparation, which can regulate the function of nervous system by reducing the secretion of aldosterone. In addition, Entresto can also reduce the accumulation of macrophages, maintain the dynamic balance of extracellular matrix, and then regulate the physiological activity of cells [22, 23]. Therefore, Entresto can make up for the deficiency of metoprolol succinate in regulating nervous system function and cell physiological activity, enhance the recovery of patients, and strengthen the therapeutic effect [23]. In line with this, our current results demonstrated that the total effective rate of the study group was higher, and after treatment, LVEF in the study group was higher. In the late 1990s, the doctors have realized that the basic mechanism of CHF is myocardial remodeling, which is the pathophysiological basis for the continuous progress of CHF [24]. When the cardiac function is damaged, the extracellular matrix and cardiomyocytes will have certain changes, and the transformation of cardiomyocytes includes cardiomyocyte apoptosis and necrosis [24]. Moreover, when the tension of the cardiovascular system is too high, the newly synthesized substances cannot divide into normal cardiomyocytes and cannot enter the normal cell cycle. If the differentiation of the cell is hindered, it may lead to compensatory growth or hypertrophy [24, 25]. According to relevant clinical trials, when the cardiac cavity is enlarged, LVEF is an independent risk factor for predicting the prognosis of CHF, which is inversely proportional to the mortality of CHF [25]. Therefore, our results suggest that Entresto combined with metoprolol succinate is effective when treating CHF and can validly enhance cardiac function.

Vascular endothelium is an important endocrine organ, which can regulate vascular tension and hematopoietic function, but when vascular endothelial function is disordered, it can accelerate the differentiation and apoptosis of endothelial cells, reduce the synthesis of NO, and then reduce its regulation of vascular tension [26]. Entresto can enhance vascular wall function by blocking local tissue RAAS activation, which can make up for the deficiency of metoprolol succinate and help patients improve vascular endothelial function [26]. The results of this study indicated that after treatment, CGRP and NO were higher, ET was lower, GSH-Px and SOD were higher, and MDA was lower compared to the control group. It is suggested that Entresto combined with metoprolol succinate could effectively strengthen vascular endothelial function and reduce oxidative stress in patients with CHF. Furthermore, Entresto can accelerate the degradation rate of enkephalin, then increase the level of NP, and promote the excretion of urine and sodium, so as to prevent cardiomyocyte fibrosis and help patients reduce myocardial injury [27]. Metoprolol succinate can not only reduce endogenous sympathetic activity but also reduce myocardial oxygen consumption, protecting cardiomyocytes [27]. Therefore, the treatment of CHF with Entresto combined with metoprolol can reduce the stress injury and reduce the oxidative stress reaction [27]. In terms of blood coagulation function, plasma prothrombin time mainly reflects the function of exogenous coagulation system, and its prolongation is mainly seen in congenital decrease of coagulation factor and fibrinogen deficiency [28]; activated partial thrombin time is mainly the examination index of endogenous coagulation factor deficiency, and its prolongation is common in hemophilia hepatopathy, DIC, and so on [29]; prolonged plasma thrombin time is common in patients with hypofibrinogenemia and abnormal fibrinemia [30]. In terms of the results of this study, the blood coagulation indexes were compared; the levels of APTT, PT, and FIB decreased; and the levels of APTT, PT, and FIB in the study group were lower compared to the control group after treatment. Our results suggest that Entresto combined with metoprolol succinate can effectively enhance the blood coagulation index, reduce blood viscosity, and further promote the clinical prognosis of patients.

Collectively, clinical practice demonstrated that LVESD and LVEDD decreased and LVEF increased after treatment with Entresto combined with metoprolol in CHF patients, which can effectively facilitate cardiac function and vascular endothelial function, reduce oxidative stress reaction, and improve blood coagulation indexes, suggesting that Entresto combined with metoprolol can improve ventricular remodeling with good safety.

## Figures and Tables

**Figure 1:** Comparison of clinical efficacy between two groups. The green bar represents the control group, and the yellow bar represents the research group.

**Figure 2:** Comparison of incidence of adverse reactions between two groups.

**Table 1:** Comparison of demographic data of two groups of patients.

Group	C group (*n* = 60)	R group (*n* = 60)	*t*/*χ*^2^	*P*
Age (years)	55.81 ± 3.53	55.83 ± 3.52	0.031	0.975
Gender (male/female)	35/25	31/29	0.538	0.462
Course of disease (year)	8.38 ± 2.11	8.39 ± 2.44	0.024	0.980
Past history				
High blood pressure	24 (40.00)	26 (43.33)	0.315	0.957
Coronary artery disease	17 (28.33)	15 (25.00)		
Diabetes	12 (20.00)	11 (18.33)		
Atrial fibrillation	7 (11.67)	8 (13.34)		

**Table 2:** Comparison of cardiac function indexes between the two groups ($\bar{x}\pm s$).

Group	*N*	LVEF (%)		LVESD (mm)		LVEDD (mm)	
		Before treatment	After treatment	Before treatment	After treatment	Before treatment	After treatment
C group	60	27.98 ± 2.44	34.81 ± 3.86^a^	46.96 ± 4.29	40.86 ± 3.14^a^	62.91 ± 4.86	56.97 ± 3.91^a^
R group	60	27.97 ± 2.45	44.86 ± 4.66^b^	46.91 ± 4.56	31.81 ± 3.92^b^	62.95 ± 4.56	43.81 ± 2.95^b^
*t*		0.022	12.865	0.061	13.957	0.046	20.811
*P*		0.982	0.000	0.950	0.000	0.963	0.000

Note: the control group before and after treatment, ^a^*P* < 0.05; the study group before and after treatment, ^b^*P* < 0.05.

**Table 3:** Comparison of vascular endothelial function between the two groups ($\bar{x}\pm s$).

Group	*N*	CGRP (ng/L)		NO (*μ*mol/L)		ET (ng/L)	
		Before treatment	After treatment	Before treatment	After treatment	Before treatment	After treatment
C group	60	11.84 ± 2.11	28.73 ± 5.38^a^	78.61 ± 4.81	90.82 ± 8.81^a^	84.83 ± 5.97	74.96 ± 4.91^a^
R group	60	11.89 ± 2.42	45.86 ± 5.83^b^	78.97 ± 4.73	113.76 ± 9.85^b^	84.98 ± 5.82	58.91 ± 5.39^b^
*t*		0.120	16.726	0.413	13.446	0.139	17.051
*P*		0.904	0.000	0.680	0.000	0.889	0.000

Note: the control group before and after treatment, ^a^*P* < 0.05; the study group before and after treatment, ^b^*P* < 0.05.

**Table 4:** Comparison of oxidative stress indexes between the two groups ($\bar{x}\pm s$).

Group	*N*	GSH-Px (U/L)		SOD (U/L)		MDA (mmol/L)	
		Before treatment	After treatment	Before treatment	After treatment	Before treatment	After treatment
C group	60	135.89 ± 9.55	235.85 ± 8.45^a^	71.92 ± 4.92	80.87 ± 5.93^a^	27.98 ± 4.56	21.87 ± 3.64^a^
R group	60	135.94 ± 9.67	365.61 ± 8.38^b^	71.93 ± 4.39	95.86 ± 4.97^b^	27.94 ± 4.49	13.19 ± 1.92^b^
*t*		0.028	84.458	0.011	15.006	0.048	16.337
*P*		0.977	0.000	0.990	0.000	0.961	0.000

Note: the control group before and after treatment, ^a^*P* < 0.05; the study group before and after treatment, ^b^*P* < 0.05.

**Table 5:** Comparison of blood coagulation function indexes between the two groups ($\bar{x}\pm \text{s}$).

Group	*N*	APTT (s)		PT (s)		FIB (g/L)	
		Before treatment	After treatment	Before treatment	After treatment	Before treatment	After treatment
C group	60	42.86 ± 3.31	37.85 ± 3.42^a^	15.73 ± 2.83	12.74 ± 1.74^a^	4.52 ± 1.22	2.79 ± 0.55^a^
R group	60	42.84 ± 3.13	32.16 ± 3.11^b^	15.48 ± 2.15	10.85 ± 1.67^b^	4.59 ± 1.34	2.01 ± 0.33^b^
*t*		0.034	9.534	0.544	6.070	0.299	9.419
*P*		0.972	0.000	0.586	0.000	0.765	0.000

Note: the control group before and after treatment, ^a^*P* < 0.05; the study group before and after treatment, ^b^*P* < 0.05.

## Data Availability

No data were used to support this study.
